# Inhibition of Reactive Gliosis Prevents Neovascular Growth in the Mouse Model of Oxygen-Induced Retinopathy

**DOI:** 10.1371/journal.pone.0022244

**Published:** 2011-07-14

**Authors:** Michael DeNiro, Falah H. Al-Mohanna, Futwan A. Al-Mohanna

**Affiliations:** 1 Research Department, King Khaled Eye Specialist Hospital, Riyadh, Saudi Arabia; 2 Department of Comparative Medicine, King Faisal Specialist Hospital & Research Centre, Riyadh, Saudi Arabia; 3 Department of Biological and Medical Research, King Faisal Specialist Hospital & Research Centre, Riyadh, Saudi Arabia; Alcon Research, Ltd., United States of America

## Abstract

Retinal neovascularization (NV) is a major cause of blindness in ischemic retinopathies. Previous investigations have indicated that ischemia upregulates GFAP and PDGF-B expression. GFAP overexpression is a hallmark of reactive gliosis (RG), which is the major pathophysiological feature of retinal damage. In addition, PDGF-B has been implicated in proliferative retinopathies. It was the aim of this study to gain insights on the possible pharmacological interventions to modulate PDGF-B and GFAP expression, and its influence on RG and NV. We used an array of assays to evaluate the effects of YC-1, a small molecule inhibitor of HIF-1 and a novel NO-independent activator of soluble guanylyl cyclase (sGC), on RG and NV, *in vivo* and *in vitro*. When compared to the DMSO-treated retinas, dual-intravitreal injections of YC-1, *in vivo*: (1) suppressed the development and elongation of neovascular sprouts in the retinas of the oxygen-induced retinopathy (OIR) mouse model; and (2) reduced ischemia-induced overexpression of GFAP and PDGF-B at the message (by 64.14±0.5% and 70.27±0.04%) and the protein levels (by 65.52±0.02% and 57.59±0.01%), respectively. In addition, at 100 µM, YC-1 treatment downregulated the hypoxia-induced overexpression of GFAP and PDGF-B at the message level in rMC-1 cells (by 71.42±0.02% and 75±0.03%), and R28 cells (by 58.62±0.02% and 50.00±0.02%), respectively; whereas, the protein levels of GFAP and PDGF-B were reduced (by 78.57±0.02% and 77.55±0.01%) in rMC-1cells, and (by 81.44±0.02% and 79.16±0.01%) in R28 cells, respectively. We demonstrate that YC-1 reversed RG during ischemic retinopathy via impairing the expression of GFAP and PDGF-B in glial cells. This is the first investigation that delves into the reversal of RG during ischemic retinal vasculopathies. In addition, the study reveals that YC-1 may exert promising therapeutic effects in the treatment of retinal and neuronal pathologies.

## Introduction

Diabetic retinopathy [DR] is a leading cause of visual disturbance in adults and is the leading cause of blindness in Americans between the ages of 20 and 74 years [1]. DR has been regarded as a retinal microvascular disease, which develops in two stages: an early, non-proliferative stage, and a later, proliferative stage. In the early non-proliferative stage, retinal vascular permeability can increase even before the appearance of clinical retinopathy [2]. Currently, this stage is diagnosed by dilation of retinal veins, retinal microaneurysmas, intraretinal microvascular abnormalities, areas of capillary nonperfusion, retinal hemorrhages, cotton wool spots, edema, and exudates. All of these signs indicate regional failure of the retinal microvascular circulation, which presumably results in ischemia. In contrast, proliferative DR's [PDR] diagnosis is based on the ischemia-induced formation of new blood vessels [BVs] on the surface of the retina. New vessels can extend into the vitreous cavity of the eye and can hemorrhage into the vitreous, resulting in visual loss [3]. They also can cause tractional retinal detachments from the accompanying contractile fibrous tissue. Furthermore, during this stage, over-proliferation of capillary endothelial cells [ECs] results in retinal neovascularization [NV], abnormal formation of new vessels in the retina and the vitreous, leading to PDR [4]. As a consequence retinal edema may ensue [5]. Retinal edema involves the breakdown of the blood-retinal barrier, with leakage of plasma from small BVs.

Platelet-derived growth factors (PDGFs) are growth-regulatory molecules that stimulate chemotaxis, proliferation, and increased metabolism of primarily connective tissue cells [6]. In addition, PDGF is a potent mitogen for mesenchymal cells and glial cells, which may act as a neuronal regulatory agent. Neuronal release of PDGF could contribute to nerve regeneration and to glial proliferation that leads to gliosis and scarring [6]. Furthermore, glial cells could utilize the elevated levels of PDGF to proliferate in RG, and under these conditions PDGF may also augment the immune responses [7]. It is also possible that PDGF increases the survival, and promotes the neurite outgrowth from grafted dopaminergic neurons [7]. PDGF-B is a vasoactive factor that possesses both chemotactic and mitogenic properties to vascular ECs *in vitro* [67] and may also have angiogenic effects *in vivo* [8]. Previous data have indicated that the distributions of PDGF B-chain-related immunoreactivity [PBRI] in the cerebral wound lesion were closely related to the NV and astrogliosis [9]. The same study has demonstrated that cerebral wound induced the expression of PDGF B-chain in neurons and macrophages in the lesion area. This increased expression of PDGF B-chain at a stab wound was proven to be related strongly to RG [9]. Moreover, increased expression of PDGF-B in the retina causes plays an important role in the pathogenesis of PDR and retinal detachment [10]. PDGF-B promotes the recruitment, proliferation and survival of pericytes; recruits glial cells [8] and retinal pigment epithelial [RPE] cells [11] that instigates scarring, which is ultimately the major cause of permanent loss of vision. Previous data have revealed that PDGF-B may play a crucial role in RG following injury [12], as well as it may lead to astrocyte and glial cell chemotaxis and proliferation [13].

The retina contains two types of macroglial cells. The most abundant are the Müller cells, which project from the retinal ganglion cell layer [GCL] to the photoreceptors. While the astrocytes, which originate in the optic nerve and migrate into the retina during development [14], reside as a single layer adjacent to the inner limiting membrane [ILM]. Glial cells provide structural and metabolic support for retinal neurons and BVs. These cells become reactive in certain injury states [15]. Several studies suggested that glial reactivity and altered glial metabolism are early pathological events in the retina during diabetes [16]. The most constant manifestation of reactivity is the increase in immunoreactivity for the intermediate filament protein [glial fibrillary acidic protein] [GFAP] [17]. GFAP is mainly expressed in astrocytes for which it constitutes a selective marker. Previous reports have demonstrated that upregulation of astrocytic intermediate filaments is a crucial step and a hallmark of RG [18]. RG is one of the pathophysiological features of retinal damage. The vertebrate retina contains a specialized type of glia, the Müller glia. Like other glial cells of the CNS, Müller cells undergo RG following acute retinal injury or chronic neuronal stress [19]. The overexpression of GFAP is the most sensitive non-specific response to retinal disease and injury, and it may be considered as the universal hallmark of retinal stress; such as retinal injury and Müller cell activation [20]. GFAP, which is located primarily in Müller cells, has specific immunoreactivities that occur in all retinal eccentricities. Moreover, virtually every pathologic alteration in the retina is accompanied by RG, that is, by distinct changes of the Müller cells properties [20]. Under these pathological conditions, Müller cells exhibit three crucial nonspecific gliotic responses, which are considered as the “hallmarks of glial cell activation”, these are: [i] cell proliferation [21]; [ii] changes in cell shape [hypertrophy] due to alterations in intermediate filament [22]; and [iii] the upregulation of the intermediate filament system composed of GFAP, vimentin, nestin and synemin [23], [24]. There are other gliotic characteristics such; targeted cellular migration [25], changes in ion transport properties [26], and secretion of signaling molecules such as VEGF [27]. Successful inhibition of GFAP using antisense oligonucleotides has also been reported by several groups [28], [29], [30]. Ostensibly, gliosis is important for the protection and repair of retinal neurons, yet some pathologies such as DR may be exacerbated by RG properties [26], [27].

YC-1; [3-[5′-hydroxymethyl-2′furyl]-1-benzyl indazole], is a small molecule that inhibits cGMP breakdown. YC-1 is an agent that has been considered as a novel type nitric oxide (NO)-independent activators of soluble guanylate cyclase (sGC) [31], [32], [33], [34]. YC-1 is not an NO donor, however, it causes activation of sGC especially in the presence of NO [35], [36], while binding to sGC at a different site from the heme [37]. We have previously shown that YC-1 suppressed retinal new vessel growth and formation in human retinal microvascular ECs, and retinal explants [38]. Furthermore, we have demonstrated that YC-1 downregulates HIF-1α, HIF-2α, VEGF, EPO, ET-1, and MMP-9 protein expression in the human retinal microvascular ECs [38], [39], [40]. The primary objectives of this investigation were to determine; [*i*] whether ischemic exposure in the OIR mouse model induces RG; [*ii*] whether YC-1 could target and hence reverse RG, and [*iii*] whether YC-1's effect is mediated through the inhibition of the length and numbers of neovascular sprouts.

## Materials and Methods

### Ethics Statement

All experiments were conducted in compliance with the laws and the regulations of the Kingdom of Saudi Arabia. In addition, all animal protocols were approved by the Institutional Review Board and conformed to the ARVO Statement for the Use of Animals in Ophthalmic and Vision Research statement of the Association for Research in Vision and Ophthalmology.” This research study was approved by the HEC/IRB Committee (Human Ethics Committee/Institutional Review Board Committee) at the King Khaled Eye Specialist Hospital (KKESH). The permit number/approval ID is “RP 0630-P”.

### Materials

YC-1 was purchased from A.G. Scientific [San Diego, CA] and dissolved in sterile dimethyl sulfoxide [DMSO]. Fluorescein isothiocyanate [FITC]-dextran 2,000,000 was purchased from Sigma-Aldrich [St. Louis, MO]. Rabbit Anti-PDGF-B polyclonal antibody was obtained from Abbiotec [San Diego, CA]. The GFAP labeling was carried out by primary rabbit-anti rat GFAP polyclonal antibody [Sigma, catalog number G9269] during immunohistochemistry; or a monoclonal GFAP antibody produced in mouse [Sigma, catalog number G3893] for Western Blot analysis. Polyclonal rabbit anti-β-actin antibody was purchased from MBL Intl [Woburn, MA].

### Tissue Culture

A transformed Müller cell line [rMC-1] was kindly sent to us by Dr. V.J. Sarthy. Müller cell cultures were grown in DMEM supplemented with 15% FBS, as well as with a fungicide mixture and 0.5% gentamicin in a humidified atmosphere of 5% CO_2_/95% air. Medium was changed every 2–3 days, and cells were grown to confluence in a 150-mm dish. Cells were split into 60-mm dishes and were used in the experiments when confluent.

R28 cells are immortalized rat retinal neurosensory/neuoroglial progenitor cells, by transfection with Adenovirus 12S E1A into the neonatal retinal tissue. The cells were a kind gift from Dr. Gail M. Seigel [SUNY, Buffalo, NY]. R28 cells express genes characteristic of neurons, as well as functional neuronal properties. R28 cells were cultured in DMEM/F12 medium in a 1∶1 mixture, supplemented with 5% FBS, 1.5 mM L-glutamine, 7.5 mM sodium pyruvate, 0.1 mM nonessential amino acids, 1× MEM, 0.37% sodium bicarbonate and 10 µg/ml gentamicin. Cells were incubated at 37°C in the presence of 5% CO_2_.

Human retinal microvascular endothelial cells [hRMVEC] were cultured in 150 µl of CS-C medium supplemented with 10% FBS and in the presence of 1–100 µM YC-1 or DMSO [0.2%] and incubated at 37°C.

### *In Vitro* Hypoxia

Cells were placed in airtight chambers [BioSpherix, Redfield, NY] and the O_2_ tension was maintained at 1.2% by using Pro-Ox Model 110 O_2_ regulator [BioSpherix, Redfield, NY]. The chamber was purged with a gas mixture of 5.32% CO_2_, and 93.48% N_2_.

### Cell Proliferation in a Co-culture System Model

To test the influence of Müller cells [rMC-1] on the hRMVECs proliferation, rMC-1 [2×10^5^ cells cm^−2^] were plated in a transwell insert [Millipore, Billerica, MA] with 0.4 mm pores and allowed to adhere overnight in 150 µL of CS-C complete medium [Cell Systems, Kirkland, WA], supplemented with 10% FBS and incubated at 37°C under normoxic [5% CO_2_/95% air]. The rMC-1 cells were then incubated under normoxic [5% CO_2_/95% air], or hypoxic conditions. To establish hypoxic conditions, cells were placed in airtight chambers [BioSpherix, Redfield, NY] that were flushed with a gas mixture of 5% CO2 and 95% N2. Oxygen concentrations within these chambers were maintained at 1.2% using Pro-Ox Model 110 O2 regulators. After treating the r-MC-1 cells with YC-1 [100 µM] for 24 hours, the insert was then placed into 24 well-plates, in which hRMVECs were plated at 5×10^3^ cells cm^−2^ and allowed to adhere overnight. hRMVECs proliferation was evaluated using 3, [4,4-dimethylthiazol-2-yl]-2,5- diphenyl tetrazolium bromide [MTT] colorimetric assay, at 24, 48, 72, and 96 hours after coculture. During the last 4 hours of each day, 100 ml of 5 mg/ml MTT [Millipore, Billerica, MA] was added in each well. Formed Formazan crystals were dissolved in 600 ml DMSO and optical density was recorded at 492 nm. Experiments were performed on at least three independent occasions. Data were presented as a percentage of negative control proliferation with **P<0.01 being significant.

### Cell Migration in a Co-culture System Model

Migration assay of hRMVECs was carried out using the transwell insert with 8 mm pore size. The inserts were coated with Extracellular matrix [ECM] [Millipore, Billerica, MA] and air-dry up. Chemotaxis was induced by the control r-MC1cells or the r-MC1 cells that were treated with YC-1 [100 µM], which were situated in the lower compartment. hRMVECs suspension [final concentration, 5×10^4^ cells/well] was added to the upper compartment. After incubated for 24 hours, the filters were washed and then fixed and stained with crystal violet [0.5% crystal violet and 20% methanol] for 30 min at room temperature. The filters were washed with distilled water, and the cells on the upper surface of the inserts were wiped with a cotton swab. The number of cells per field that migrated to the lower surface of the filters was determined microscopically. Five randomly chosen fields were counted per filter. Data were presented as a number of migrated cells [**P<0.01].

### Quantitative RT-PCR by Molecular Beacon Assays

The message levels for *PDGF-B* and *GFAP* were quantified by Real time RT-PCR. Gene-specific molecular beacons and primers were designed to encompass the genes of interest, with beacon's annealing site to overlap with the exon-exon junctions for additional specificity [Beacon Designer 6.0, Premier Biosoft International, Palo Alto, CA, USA]. Threshold cycle [Ct] values for the different samples were utilized for the calculation of gene expression fold change using the formula 2 to the minus power of delta delta ct. Fold changes in the *PDGF-B* and *GFAP* gene relative to the *β-actin* endogenous control gene were determined by the following equation: fold change = 2^−Δ [Δ*C*^_T_^]^, where change in threshold cycle [Δ*C*_T_] = *C*_T_ [*gene of interest*]−*C*_T_ [*β-actin*] and Δ [Δ*C*_T_] = Δ*C*_T_ [treated]−Δ*C*_T_ [untreated].

### Western Blot

Müller cells [rMC-1] and R28 cells were seeded overnight in 6-well plates [3×10^5^ cells/well]. Cells were treated with either YC-1 [25–100 µM] or DMSO [0.2% *v/v*] for 72 hours under normoxic or hypoxic environments. Reactions were terminated by addition of lysis buffer [Cell Signaling, Beverly, MA]. Protein content of the cell lysates was determined according to the Bradford method [Bio-Rad, Hercules, CA]. Aliquots [40 µg] of whole-cell lysates were separated on 7.5% SDS-PAGE, and electro-transferred onto polyvinylidene membranes [Amersham Pharmacia Biotech, Little Chalfont]. After blocking with 5% nonfat dry milk in TBS-T, the blots were incubated overnight with anti-[GFAP, PEDG-B, and β-actin (internal control)] antibodies. Then blots were washed 3×10 min washes in PBS/tween and subsequently incubated with peroxidase-conjugated anti-mouse IgG secondary antibody at 1∶3000. The signals were obtained by enhanced chemiluminescence [Amersham Biosciences], and visualized by exposure to X-ray film. Upon completion of chemiluminescence, equal lane loading was checked by Ponceau S Solution [Sigma, St. Louis, MO]. X-ray films were scanned with a computer-assisted densitometer [model G-710; Bio-Rad] to quantify band optical density [Quantity One software; Bio-Rad].

### GFAP Immunofluorescence

Müller cells [rMC-1] and R28 cells [2×10^4^ cells per well] were grown on 8-well chamber slides and cultured in 300 µl of their growing media, which contained YC-1 [25–100 µM] or DMSO [0.2% *v/v*] and incubated under normoxia or hypoxia for 48 hours at 37°C. YC-1 or DMSO was added 5 minutes prior to the hypoxic incubation. Immunofluorescence of rMC-1 and R28 cells was conducted by blocking slides in 0.1% blocking solution (Invitrogen/Molecular Probes TSA Kit #2: T-20912) followed by incubation for two hours with the primary rabbit-anti rat GFAP polyclonal antibody [Sigma, catalog number G9269], diluted in 0.1% blocking solution in a humid chamber for 2 hours at 4°C. Negative controls included omission of the primary antibody or its substitution with phosphate-buffered saline (PBS). This was followed by incubating the slides with the horseradish peroxidase (HRP)-labeled goat anti-rabbit IgG (H+L) secondary antibody (#A-11008) in conjunction with a dye-labeled tyramide [AlexaFluor 488] (Invitrogen/Molecular Probes Carlsbad, California] [TSA Kit #2] for 1 hour in a dark humid chamber at room temperature. These processes results in localized deposition of the activated tyramide derivative (Stage 1). Hence, further dye deposition, and therefore higher levels of signal amplification, can be generated by detecting dye deposited in “Stage 1” with a horseradish peroxidase (HRP)-labeled anti-dye antibody in conjunction with a dye-labeled tyramide “Stage 2”. Immunofluorescence was visualized by using a Zeiss microscope [Zeiss LSM 510 META inverted confocal microscope equipped with argon and helium/neon lasers using excitation wavelengths 488, on Axiovert 200 M, Thornwood, NY]. Digitized images were acquired utilizing excitation wave length 488 nm. Intensity values of immunofluorescence staining of GFAP in rMC-1 and R28 cells was analyzed and quantified using Metamorph™ imaging analysis software version 6.0 [Universal Imaging, Sunnyvale, CA]. The staining intensity in our series ranged from a weak blush to moderate or strong. The amount of cells staining with the antibody was further categorized as focal [<10%], patchy [10%–50%], and diffuse/multifocal [>50%]. For semiquantitative analysis, focal and/or weak staining was considered equivocal staining, and patchy or diffuse/multifocal staining was subcategorized as either moderate or strong.

### Animals and Experimental Design

C57BL/6J mice, from Jackson Laboratory [Bar harbor, ME] were used in these experiments. All animal protocols were approved by the Institutional Review Board and conformed to the ARVO Statement for the Use of Animals in Ophthalmic and Vision Research statement of the Association for Research in Vision and Ophthalmology. Mice were divided into four separate groups; [1] Non-treated mice grown under ambient conditions [negative control]; [2] non-treated hyperoxia-exposed mice [positive control]; [3] DMSO- treated hyperoxia-exposed mice [sham-treated]; and [4] YC-1-treated hyperoxia-exposed mice [drug-treated].

### Mouse Model of Oxygen Induced Retinopathy

Retinal NV was induced in newborn mice as described previously [41]. Briefly, P7 mice were exposed with their nursing mother, for 5 days [between P7 and P12] to hyperoxic conditions, by incubating them in an airtight chamber [PROOX 110 chamber O_2_ controller; Biospherix Ltd., Redfield, NY] ventilated by a mixture of O_2_ and air to a final oxygen fraction of 75±2%. These incubation conditions induced vaso-obliteration and subsequent cessation of vascular development in the capillary beds of the central retina [41]. At P12, the mice were allowed to recover in normal room air conditions and maintained for another 5 days [till P17], the day in which peak disease occurs. A condition of relative hypoxia resulted between P12 and P17, and extensive retinal NV developed in 100% of the mice. Age-matched animals with the hyperoxia-exposed groups were maintained identically, except they were exposed to room air [21% O2, 79% N2] for the duration of the experiment. Animals were examined and sacrificed on the same days.

### Intravitreal Drug Injections

A group of hyperoxia-exposed animals [n = 15] were injected intravitreally [into both eyes] at P12 and P15 with 3 µl of YC-1 [100 µM] [drug-treated group]. Another group of hyperoxia-exposed mice [n = 15] were injected intravitreally [into both eyes] at P12 and P15 with 3 µl of DMSO [0.2% (v/v)]. Non-treated mice grown under ambient conditions, non-treated hyperoxia-exposed mice, DMSO- treated hyperoxia-exposed mice and YC-1-treated hyperoxia-exposed mice, were all examined at different critical time points for qualitative assessment of the retinal vasculature by fluorescein angiography.

### Retinal Fluorescein Angiography and Visualization of Retinal Vascularization

Deep anesthesia was induced by intraperitoneal injection of ketamine [1%], xylazine [0.1%], and sodium chloride [0.9%] in a concentration of 0.1 mL/10 g mouse body weight. Sternotomy was performed, the mice were perfused through the left ventricle with 600 µL of high-molecular-mass [2×10^6^ Da] FITC-dextran in PBS [50 mg/ml], which was allowed to circulate for 2 minutes before the animals were euthanatized and the eyes enucleated and the flat mounts were prepared. Subsequent to retinal extraction, all retinas were fixed in 4% paraformaldehyde for 24 hrs at 4°C. A dissecting microscope was used to dissect the cornea with a circumferential limbal incision, followed by removal of the lens and vitreous. Microscissors were used to make four radial incisions of the retinal eyecup in order to prepare retinal flat mounts on glass slides. Flat mounts were immersed in Aquamount mounting medium [Polysciences, Warrington, PA], coverslips were placed over the retina, and the edges of the coverslips were sealed.

### Immunohistochemistry

Mouse retinas were dissected and prepared for immunohistochemical analysis, fixed in 4% paraformaldehyde in 0.1 M PBS for 15 min at room temperature and embedded in paraffin, sectioned [5 µm]. Tissue sections were deparaffinized, hydrated, and later exposed to heat-induced antigen retrieval using a microwave oven [three 5-minute cycles in citrate buffer, pH 6.0], endogenous peroxidase was abolished with methanol, and hydrogen peroxide and nonspecific background staining was blocked by incubating the tissue sections for 5 minutes in normal swine serum. Subsequently, all slides were washed three times in PBS, and incubated for 1 hour with primary anti–[PDGF-B, GFAP, and β-actin] antibodies. The sections were washed with TBST and incubated with EnVision Polymer HRP secondary antibody [DAKO, Carpinteria, CA] for 30 minutes. All slides were stained with DAB solution and counterstained with hematoxylin. Slides were cover slipped [Permount; Fisher Scientific, Fairlawn, NJ] and examined by light microscopy. Negative controls included omission of the primary antibody or its substitution with phosphate-buffered saline (PBS). Sections were photographed under a microscope [Zeiss Axiovert 135, Thornwood, NY], and images were acquired a digital camera [AxioCam, NY]. All retinas were examined at ×60 objective. The staining intensity in our series ranged from a weak blush to moderate or strong. The amount of cells staining with the antibody was further categorized as focal [<10%], patchy [10%–50%], and diffuse/multifocal [>50%]. For meaningful semiquantitative analysis, focal and/or weak staining was considered equivocal staining, and patchy or diffuse/multifocal staining was either subcategorized as either moderate or strong staining. All Immunohistochemical analyses were measured by Metamorph digital image software [Molecular Devices, Sunnyvale, CA].

### Quantitative Image Analysis of Immunohistochemical Staining

GFAP and PDGF-B positive immunostaining in retinal tissue sections (immunohistochemistry), as well as GFAP positive immunolabeling in rMC-1 and R28 cells (immunocytochemistry), were all visualized and captured using AxioCam digital microscope camera. The filter was set with excitation wavelengths 488. MetaMorph image analysis software (version 7.1, Universal Imaging, Downingtown, PA) was used for image processing and quantitative analysis of GFAP and PDGF-B positive immunostaining. MetaMorph tools were used to set the threshold and regions of interest (ROIs). All images were captured at identical time and exposure settings, and they were all processed to the same scale. Images were first segmented on the basis of pixel intensity, which was done on a plane-by-plane basis for an image stack. Briefly, each retinal section was scanned into Metamorph, and five (5) fields/slide were chosen from each section for analysis. One hundred and fifty (150) cells from each field were selected. The saved file was used to calibrate each image for specific pixel size. With the help of a free drawing tool, GFAP and PDGF-B-stained areas were chosen and measured in total-pixels area. A threshold encompassing an intensity range of 100–250 gray-scale values was applied to the ROIs in the least brightly stained condition first. The data were also read and investigated by Matlab v6.5 script file software, which counted the total number of pixels that were above threshold value. This number was divided by the total number of pixels in each image to yield percent fluorescent pixels. To correct for background fluorescence, the threshold was adjusted for each experimental series, with concomitantly processed negative controls used as the guide for setting background fluorescence. The background fluorescence intensities per pixel were subtracted from the experimental data by using a one-step erosion procedure, and then all remaining objects were counted. The same threshold was subsequently applied to all images. GFAP and PDGF-B was considered to be positive only when it exceeded the established threshold. Percent GFAP and PDGF-B expression above threshold in the total area selected was then calculated. The total GFAP and PDGF-B fluorescence intensity per cell was calculated, and the average fluorescence intensity per pixel was determined by dividing the total intensity by the area of the cell measured in pixels. This was followed by measuring the average fluorescence intensity in each field. Data from multiple fields as indicated over several experiments were used to obtain the final results. The number of immunopositive-stained cells per image was then expressed per um^2^, and the average number per section was determined among five separate fields.

### Statistical Analysis

Analysis was performed utilizing ANOVA for multiple variables and with *t*–Tests for comparison of 2 groups with normal distribution. For the analysis of Real Time RT-PCR data; immunohistochemistry data; Western Blot data, analysis was performed with ANOVA for multiple variables and with *t*–Tests. Data are expressed as mean ± SEM from at least 3 independent experiments. Significance was defined as *P<0.05; **P<0.01; ***P<0.001.

## Results

### Analyses of the Retinal Vasculature and the Progression of Retinal NV

At P2 only budding superficial vessels were observed occupying a single plane around the optic disc [Fig. 1; P2]. In P4 wild type mice, the retinal vasculature was organized uniformly and was evenly spaced over the superficial retina and vessels grew into the deeper layers of the retina [Fig. 1; P4]. The vascular density and the number of branch-surrounded spaces increased at P4. In addition, the margin of the developing BVs on the surface of the retina is located halfway between the optic nerve and the peripheral edge of the retina. This is followed by development of a capillary network at P7. During P7, superficial vessels cover about 80% of the retina [Fig. 1; P7]. At this stage sprouts from superficial vessels begin to grow into the retina to form the intermediate and deep capillary beds. In addition, the hyaloidal vessels start to regress. Over the course of the next week, the primary superficial network extended toward the periphery, reaching the far periphery at P12. Angiogram of P12 FITC-dextran-perfused retinal flat mounts of the OIR model preparations displays the effects of 5 days of hyperoxic-exposure [Fig. 1; P12]. On return to normoxia at P12, a relative state of ischemia in the poorly vascularized retina is associated with the excessive re-growth of superficial vessels, leading to abnormal sprouting at the interface between retina and vitreous. Retinas at P12 exhibit typical signs of central non-perfusion of the retina and a drastic regression in the vascular network, leaving only the major vessels and practically no capillary network. The peripheral retina still showed evidence of a vascular network, but, in general, the deep vascular plexuses had completely failed to form. By P15 the retinal ischemia initiates an aggressive neovascular response at the interface of the perfused retinal periphery and the ischemic central capillary beds [Fig. 1; P15]. On P17, the vascular network of the O2-injured retinas was significantly altered as demonstrated by an increase in retinal NV. These retinas displayed the features indicative for a strong ongoing vasoproliferative response: central capillary-free regions, vessel tortuosity and BV tufts [Fig. 1; P17].

**Figure 1:** Analyses of Retinal Vascular Development in the Normal Retinal Vasculature and the Neovascular Retina. Mice were perfused with fluorescein-labeled dextran. Normal mice were analyzed P2 [A], P4 [B], and P7 [C]. Exposure of mice to 75% O_2_ between P7–P12 led to rapidly progressive vaso-obliteration of the retinal vasculature over. Retinal NV was analyzed in the OIR mice on P12 [D], P15 (OIR) [E], and P17 (OIR) [F]. [n = 15 per group]. bar: 300 µm.

### YC-1 Attenuates Neovascular Sprouting in the OIR Mouse Model

Data from [Figs. 2A–F] demonstrated that retinal NV in the O_2_-injured and the DMSO-treated retinas was associated with the presence of neovascular sprouts and the formation of cordlike or tube-like structures. However, YC-1 treatment has disturbed and suppressed the development and elongation of neovascular sprouts [Figs. 2C–F]. YC-1 significantly and dose-dependently reduced the total length [Fig. 3A] and the number [Fig. 3B] of neovascular sprouts, as compared to DMSO-treated retinas.

**Figure 2:** The Influence of YC-1 on Neovascular Sprouts Number and Length. Images exhibit a higher magnification of growing tips of BVs that reveal multiple neovascular sprouts growing at multiple angles including both along and above the plane of the section. Image along the leading edge of vascularization from; [A] Non-treated ischemic retinas; [B] DMSO-treated retinas; [C, D, E, and F] represent retinas from animals that were injected with YC-1 [25–100 µl]. neovascular sprouts lengths and numbers were not influenced by DMSO treatment. Whereas treatment with YC-1 significantly and dose-dependently inhibited the number and the length of neovascular sprouts. [n = 5 per group].

**Figure 3:** YC-1 Reverses Retinal Reactive Gliosis and Retinal Neovascularization, *in vivo* and *in vitro*. Neovascular sprouts from DMSO-treated retinas had approximately similar lengths as the non-treated ischemic retinas [A]. YC-1 treated animals exhibited a significant and a dose-dependent decrease in neovascular sprouts lengths as compared to DMSO-treated retinas. [ANOVA, ***P<0.001; **P<0.01 between YC-1 and DMSO] [A]. DMSO has no influence on the number of neovascular sprouts [B]. Whereas YC-1 exhibited a significant and a dose-dependent decrease in neovascular sprouts number [B]. [ANOVA, ***P<0.001; **P<0.01 between YC-1 and DMSO]. There were 24 neovascular sprouts/retina that were averaged. [n = 5 per group]. By using primer sets [C]; Real Time RT-PCR analyses, *in vivo* [D and E] indicate that the levels of *GFAP* and *PDGF-B* mRNA were increased in the non-treated ischemic retinas, while non-treated normoxic retinas exhibited extremely low levels. Treatment of ischemic retinas with dual injections of YC-1 resulted in a significant knockdown of PDGF-B [**P<0.01] and GFAP [**P<0.01] gene expression when compared with DMSO-treated controls. ANOVA; Mean ± SEM of mRNA level normalized to β-actin were calculated, [***P<0.001 and **P<0.01, as compared to DMSO-treated retinas]. Data are representative of 3 independent experiments. Real Time RT-PCR analysis, *in vitro* [F] indicate that post-culturing R28 and rMC-1 cells under normoxic and hypoxic conditions; the mRNA levels of *GFAP and PDGF-B* were upregulated in all non-treated hypoxic cells, while normoxic cells exhibited remarkable low mRNA levels. Treatment of hypoxic R28 and rMC-1 cells with various concentrations of YC-1 resulted in a significant inhibition of *GFAP and PDGF-B*, mRNA expression as compared to DMSO-treated controls. ANOVA was used for statistical analyses. Mean ± SEM of mRNA level normalized to β-actin were calculated, [***P<0.001 and **P<0.01 as compared to DMSO-treated hypoxic control. Data are representative of 3 independent experiments].

### YC-1 Reverses Retinal Reactive Gliosis and Retinal Neovascularization, *in vivo* and *in vitro*

In order to investigate the mechanisms via which YC-1 reverses retinal RG and NV in the OIR mouse model, we measured the transcription of key genes that are associated with both; RG and NV, as markers of a putative recovery. By using the primers, which were summarized in [Fig. 3C]; Real Time RT-PCR data have indicated that there was a significant enhancement of *GFAP* gene expression levels in the non-treated ischemic retinas as compared with the retinas from animals that were placed under ambient conditions. The effects of DMSO-treatment on the gene expression profiles paralleled those seen in the non-treated ischemic retinas. YC-1 treatment significantly attenuated [**P<0.01] the message levels of *GFAP* expression [Fig. 3D]. YC-1 treatment [100 µM] reduced ischemia-induced overexpression of GFAP at the message [by 64.14±0.5%], as compared to DMSO-treated controls. Furthermore, there was a significant alteration in the mRNA levels of PDGF-B, between YC-1-treated groups and non-treated and DMSO-treated controls. There was a significant upregulation in the mRNA levels of *PDGF-B* in the ischemic retina as compared to normoxic retinas [Fig. 3E]. Treatment of the animals with YC-1 [100 µM] significantly [**P<0.01] attenuated the ischemia-induced overexpression of *PDGF-B* at the message level of [by 70.27±0.04%], as compared to DMSO-treated retinas.

Our *in vitro* studies have revealed that post hypoxic exposure, the level of *GFAP* mRNA expression was significantly increased over the normoxic control, which displayed a basal expression levels [Fig. 3F]. The effects of DMSO-treatment on the gene expression patterns in both cell types paralleled those seen in the non-treated ischemic retinas. Treatment of r-MC1 and R28 cells with 25–100 µM YC-1 resulted in significant dose-dependent attenuations in the message levels of *GFAP* expression, when compared with DMSO-treated hypoxic cells. At 100 µM, YC-1 treatment downregulated the hypoxia-induced overexpression of *GFAP* at the message level in rMC-1 cells [by 71.42±0.02%], and R28 cells [by 58.62±0.02%], respectively. Data were normalized to β-actin mRNA levels. In addition, Real Time RT-PCR data have demonstrated that after 48 hours of hypoxic exposure, the levels of *PDGF-B* mRNA expression were significantly increased over the normoxic control, which displayed low gene expression levels [Fig. 3F]. Treatment of both cell lines YC-1 [25–100 µM] resulted in significant dose-dependent attenuations in the message levels of *PDGF-B* expressions, when compared with DMSO-treated hypoxic cells. Treatment of r-MC1 and R28 cells with YC-1 at 100 µM downregulated the hypoxia-induced overexpression of PDGF-B at the message level in rMC-1 cells [by 75±0.03%], and R28 cells [by 50.00±0.02%], respectively.

### Immunohistochemical Expression and Localization of PDGF-B, and GFAP, *in vivo*

In the *Non-Treated Normoxic Retinas* [Fig. 4], PDGF-B expression was focal and sparse, and it was predominantly localized in the ILM, NFL, GCL, and INL. Furthermore, the *Non-Treated Ischemic Retinas* exhibited a pattern of PDGF-B overexpression and immunohistolocalization, which was particularly prominent in the ganglion cells [GCL], as well as a significant upregulation in the positive immunoreactivities of PDGF-B, which was present in the ILM, and within the NFL, and the inner segments of the photoreceptor cells [INL]. The immunoreactivity was diffuse with strong PDGF-B overexpression that was primarily augmented in the NFL, GCL, and INL, as compared to *Nontreated Normoxic Retinas* and the *YC-1-Treated Retinas*. In the *DMSO-Treated Retinas*, the immunohistolocalization pattern of PDGF-B was identical to the pattern that was shown in the ischemic controls. In the YC-1-treated retinas; PDGF-B immunoreactivity was significantly inhibited [by 57.59±0.01%], as compared with DMSO-treated retinas, and the immunostaining was primarily focally localized in the ILM, GCL, and INL [Fig. 4].

**Figure 4:** Immunohistochemical Analysis of PDGF-B, *in vivo*. Photomicrographs of retinas from various OIR groups that were immunostained for PDGF-B. The expression of PDGF-B was upregulated in the non-treated ischemic and DMSO-treated groups, compared with non-treated normoxic group. While all protein immunoreactivities were downregulated in the YC-1-treated group, compared with DMSO-treated groups. Data are representative of 3 independent experiments. Scale bar: 140 µm.

Our immunohistochemistry data have demonstrated that the *Nontreated Normoxic Retinas* exhibited staining signals for GFAP immunoreactivity, which tended to be sparse and focal and primarily localized in the ILM and GCL [Fig. 5]. However, the *Nontreated O_2_-Injured* and the *DMSO-Treated O_2_-Injured Retinas* exhibited strong staining of GFAP expression, primarily in the ILM, nerve fiber layer [NFL], GCL, and inner nuclear layer [INL] of the ischemic retinas. In addition, there was a strong staining for GFAP immunoreacreactivity in Müller cell processes throughout the retina. In contrast, *YC-1-Treated retinas* displayed a significant downregulation in GFAP immunoexpression as compared to *DMSO-Treated Retinas* [Fig. 5]. in addition, GFAP expression was weak “focal”, sparse, sporadic and primarily localized in the ILM, NFL, and the GCL regions of these retinas. Our data has indicated that YC-1 treatment [100 µM] has reduced ischemia-induced overexpression of GFAP protein levels [by 65.52±0.02%], as compared to *DMSO-Treated Controls* [Fig. 5].

**Figure 5:** Immunohistochemical Analysis of GFAP, *in vivo*. Photomicrographs of retinas from OIR groups that were immunostained for GFAP. GFAP was overexpressed in the non-treated ischemic and DMSO-treated groups, compared with non-treated normoxic group. Whereas all GFAP immunoreactivities were downregulated in the YC-1-treated group, compared with DMSO-treated groups. Data are representative of 3 independent experiments. Scale bar: 140 µm.

Our data analysis of PDGF-B and GFAP expression in the retinal tissues indicated that YC-1 significantly reduced the number of PDGF-B (+) cells and GFAP (+) cells as compared to DMSO-treated retinas [Fig. 6A], which indicated that YC-1 exhibited anti-reactive gliosis and anti-angiogenic properties, *in vivo*.

**Figure 6:** YC-1 Exhibits Anti-Reactive Gliosis and Anti-Angiogenic Properties, *in vivo* and *in vitro*. Assessments of retinal immunohistochemical analysis exhibit the values that were obtained from at least 5 retinal fields were used to calculate the average pixel intensity value/retina [A]. Bar graphs exhibit the area of staining of GFAP and PDGF-B in all four groups. Values [mean ± SEM], from 3 separate experiments from at least 10 images from 4 different eyes/group. [***P<0.001 and **P<0.01 as compared to DMSO-treated retinas]. [B] Coculture models. [*i*] Cell proliferation assay model. [*ii*] Cell migration assay model; were both utilized to investigate the effects of YC-1 on the proliferation [C] and migration [D] of ECs in a coculture system. hRMVECs growth curves from four groups were depicted. Coculture group had a higher proliferation and migration rate of hRMVECs cells than that of hRMVECs solo [**P<0.01]. Hypoxia significantly increased hRMVECs proliferation and migration rate in the coculture system [**P<0.01, rMC-1/hypoxia vs. rMC-1/normoxia]. After rMC-1 cells were treated with YC-1 [100 µM], the proliferation and the migration rate of hRMVECs were significantly inhibited compared with the rMC-1/hypoxia group. [**P<0.01, YC-1-treated rMC-1/hypoxia vs. nontreated rMC-1/hypoxia]. Data are representative of 3 independent experiments.

### Inhibition of ECs Proliferation and Migration in the Coculture System via the Anti-angiogenic Effects of YC-1 on Müller Cells

Our proliferation assay in a coculture system model has demonstrated that rMC-1cells-hRMVECs coculture significantly increased hRMVECs proliferation compared to solo hRMVECs culture [Fig. 6B and 6C] under normoxia and hypoxia. Data have indicated that coculture under hypoxic conditions had a synergistic effect. Although there was insignificant difference in the hRMVECs proliferation while being cocultured with nontreated rMC-1 cells under normoxic or hypoxic conditions; the proliferation of hRMVECs was significantly suppressed when rMC-1 cells were treated with YC-1, under normoxic and hypoxic conditions. Furthermore, our migration assay in a coculture system model has shown that hRMVECs were found to extend through 8.0 mm Transwell pores in a transmigration assay with Müller cells grown in the well [Fig. 6C and 6D]. Coculture of hRMVECs with Müller cells under hypoxia resulted in a significant increase in hRMVECs migratory activity over the levels of [rMC-1 cells/normoxia group]. Whereas the rMC-1 cells-induced hRMVECs migration was significantly attenuated by YC-1 treatment under normoxic [rMC-1 cells/hRMVECs (normoxia group)] and hypoxic conditions [rMC-1 cells/hRMVECs (hypoxia group)] [Fig. 6C and 6D].

### YC-1 Restrains Hypoxia-Induced Upregulation of GFAP and PDGF-B Protein Levels, in Glial Cells

In order to investigate the mechanisms via which YC-1 reverses retinal RG and NV in our cell culture models, we quantified the expression of GFAP and PDGF-B, respectively, as key protein molecules that are associated with RG and NV. Our Western immunoblot data have indicated that rMC-1 and R28 cells cultured under normoxia exhibited suppressed protein levels of GFAP protein, whereas GFAP was overexpressed 72 hours post-hypoxic exposure [Fig. 7A]. In the DMSO-treated hypoxic cells, GFAP protein expression remained relatively stable, when compared with non-treated hypoxic cells. This increase in GFAP expression was measured by densitometry [Fig. 7B]. In both cell types and under hypoxic conditions; YC-1 treatment dose-dependently inhibited the hypoxia-induced GFAP protein levels in by [78.57±0.02%] in rMC-1cells, and by [81.44±0.02%] in R28 cells, respectively. Furthermore, Western immunoblot analysis have indicated that rMC-1 and R28 cells cultured under normoxia exhibited low immunoreactivity signals of PDGF-B protein expression, while this signal was overexpressed after 72 hours of hypoxic exposure [Fig. 7A]. There was a significant increase in PDGF-B protein expression, as measured by densitometry [Fig. 7B], compared to normoxia. In both cell types and under hypoxia, YC-1 inhibited the hypoxia-induced upregulation of PDGF-B protein levels in a dose-dependent manner, compared with DMSO-treated hypoxic cells. At 100 µM, YC-1 treatment inhibited the hypoxia-induced protein overexpression of PDGF-B [by 77.55±0.01%] in rMC-1cells, and [by 79.16±0.01%] in R28 cells, respectively.

**Figure 7:** YC-1 Restrains Hypoxia-Induced Upregulation of GFAP and PDGF-B Protein Levels, in Glial Cells. Western Blot analysis indicated that protein expression levels were elevated markedly in the non-treated hypoxic cells [A]. In YC-1-treated hypoxic cells, GFAP and PDGF-B protein expression were significantly decreased in a dose-dependent fashion, compared with DMSO-treated hypoxic cells. Statistical significance was determined by ANOVA [**P<0.01]. Data are representative of 3 independent experiments. The densitometric analysis of Western Blot data [B] represents the intensities of GFAP and PDGF-B protein expressions in rMC-1 and R28 cells relative to those of β-actin expression, whereas the relative ratio of hypoxia control was defined as 100. Values, shown as the mean ± SEM, from 3 separate experiments with a total sample size of 6. [**P<0.01 as compared to DMSO-treated hypoxic control].

Our immunofluorescence staining of GFAP demonstrated that non-treated rMC-1 and R28 cells cultured under hypoxia displayed enriched GFAP protein fluorescence immunoreactivity, with strong cytoplasmic staining of both cell types [Fig. 8; positive control]. Hypoxic cells exhibited significant (**P<0.01) increase in GFAP protein levels, as compared with normoxic cells, which exhibited limited areas of very weak “blush” GFAP staining [Fig. 8; negative control]. Furthermore, there was a strong positive GFAP staining signal deposited over the cytoplasms of the DMSO-treated cells cultured for 48 hours under hypoxia [Fig. 8; DMSO]. This intense positive staining was diminished with YC-1 treatment. No GFAP staining was observed in experiments in which the primary antibody was omitted and/or substituted with PBS (data not shown). rMC-1 cells treated with 25 µM YC-1 displayed the presence of cytoplasmic localization but then with weaker equivocal “weak” staining intensity. Whereas, a stronger diffuse cytoplasmic GFAP staining was observed in R28 cells. Treatment of rMC-1 and R28 cells with 25 µM YC-1 under hypoxia for 48 hours displayed a significant inhibitory effects (42.10% and 48.78% inhibition, respectively), compared to DMSO-treated hypoxic controls. At 50 µM YC-1, GFAP cytoplasmic staining levels was drastically reduced in both cell types, as compared with non-treated controls cultured under hypoxia. At [50 and 75 µM], YC-1 had significant inhibitory effects on GFAP protein expression in both cell types, as compared to hypoxic controls. There was a strong reduction of GFAP cytoplasmic staining levels in both cell types, as compared with non-treated controls cultured under hypoxia. Treatment of rMC-1 and R28 cell lines with 50 µM YC-1 for 48 hours under hypoxia, caused a significant inhibition of 44.73% (**P<0.01) and 50% (*P<0.05) respectively, as compared with non-treated hypoxic controls. Whereas treatment of cells with 75 µM YC-1 for 48 hours under hypoxic conditions had significant (**P<0.01) down-regulatory effects on GFAP protein expression in both cell types, whereas GFAP inhibition in rMC-1 and R28 cells were 52.63% and 56.09%, respectively, as compared with non-treated hypoxic controls. At 100 µM YC-1, there were few stained regions that were still detected in the cytoplasm of YC-1-treated cells. At 100 µM, YC-1 displayed significant (**P<0.01) 78.94% and 70.73% folds of inhibition in rMC-1 and R28 cells, respectively, as compared with non-treated hypoxic controls. Our data indicated that YC-1 significantly reduced GFAP protein levels in R28 and rMC-1 cells under hypoxia and in a dose-dependent fashion [**P<0.01] [Fig. 8 and bottom graphs in Fig. 8].

**Figure 8:** Immunofluorescence Analysis of GFAP Expression, *in vitro*. Photomicrographs show the rMC-1 and R28 cells, which were immunostained with anti-GFAP antibody. Intense staining was considered a positive signal. Yellow arrows indicate GFAP immunostaining. Under hypoxia, non-treated hypoxic cells exhibited extremely high GFAP immunoreactivity. Treatment of cells with YC-1 [25–100 µM] under hypoxia for 48 hours resulted in a dose-dependent inhibition of GFAP expression. Images are representatives of 3 independent experiments. Scale bar: 40 µm. Graphs in the bottom represent the assessments of the cellular immunocytochemical analysis of GFAP. Graphs showing the intensity of GFAP staining in rMC-1 and R28 cells after treatment with YC-1 relative to that measured in DMSO-treated hypoxic control. The areas of staining to GFAP/µm^2^ in all four groups were measured. Values, shown as the mean ± SEM, from 3 separate experiments.

## Discussion

Reactive gliosis [RG] is one of the pathophysiological features of retinal damage. RG includes morphological, biochemical, and physiological changes of Müller cells; these alterations vary with type and severity of damage. The molecular mechanism(s) leading to RG is not fully elucidated. In this study we have investigated the effects of YC-1, a small molecule inhibitor of hypoxia induced factor -1 (HIF-1), on experimentally induced retinopathy using the OIR mouse model. YC-1 is a novel type nitric oxide (NO)-independent activators of soluble guanylate cyclase (sGC) [31], [32], [33], [34]. YC-1 is not an NO donor, however, it causes activation of sGC especially in the presence of NO [35], [36], while binding to sGC at a different site from the heme [37]. Data has previously demonstrated that sustained hyperoxia effectively preserved astrocytes in the central retina in spite of extensive damage to the capillary networks and prevented the reactive expression of GFAP in the Müller glia [42]. In addition, the OIR mouse model has been extensively used because it constitutes several clinical manifestations that are analogous to the retinopathy of maturity [ROP], and mimics the important aspects of PDR; the most common ischemic retinopathy in patients [43]. Since (i) YC-1 induces physiological RV in the OIR model [39]; (ii) a significant segment of this process seems to occur in the INL, OPL, ONL, and OLM retinal cell layers; and (iii) the fact that Müller cells processes span the entire retina and extend from the INL to the OLM, the possibility existed that YC-1 maybe acting directly on retinal glial cells. We found that GFAP [the hallmark of RG] was expressed at low levels under normoxic conditions, *in vitro* and *in vivo*, which is in concordance with what's been previously reported [44]. However, upon exposure to hypoxic/ischemic conditions, GFAP levels were increased both at the message and the protein levels. These results are in agreement to what has been previously reported by other studies, which indicated that hypoxic subculture of Müller cells causes a dramatic upregulation of GFAP *in vitro* [45]. Retinal ischemia/hypoxia have been shown to cause an increase in gene and protein expression of GFAP in Müller cells within 1–3 h and that expression extended the inner processes of Müller cells [up to the INL] [46], [48]. It has been noted that astrocytes are the only cells in the retina that express GFAP, but after various insults such as retinal detachment, ischemia, light damage, or genetic photoreceptor degeneration, Müller glia become GFAP-positive [49], [50], whereas *Normoxic Retinas* expressed low levels of GFAP expression that was confined to the ILM and GCL regions of the retina, with no Müller cell processes staining. In the *Nontreated Ischemic Retinas* and *DMSO-Treated Ischemic Retinas*; GFAP was significantly upregulated in the ILM, GCL, IPL, and INL with clear staining at Müller cell processes, and was overly expressed due to the damage to the retina by ischemia after vascular pruning, which indicates glial reactivity.

YC-1 displays antiangiogenic activities *in vitro* and *in vivo* [38], [39], [40]. YC-1 possesses novel pleiotropic effects pertaining the making, toning, maintaining the structural and functional integrities of BVs. Our results show that YC-1 repressed GFAP expression at the message and the protein levels, in the ischemic retinas and in glial cells, suggesting a reversal of RG. To our knowledge no other report to date has demonstrated the ability of small anti-angiogenic molecules to target and reverse RG.

Previous studies have demonstrated that levels of PDGF-B were increased after ischemic injury [51]. Since YC-1 inhibits platelet aggregation, it is plausible that some of its anti-angiogenic effects in retinal vasculopathies are mediated through PDGF-B. Our data demonstrate that under hypoxic conditions PDGF-B is expressed at significantly higher levels compared to normoxic retinas. YC-1-treated retinas exhibited a significant inhibition of PDGF-B mRNA and protein levels as compared to DMSO-treated retinas. It is noteworthy that other groups have attributed the retinal production of PDGF-B to the ganglion cells [52]. Our data indicated *Nontreated Ischemic Retinas* and *DMSO-Treated Ischemic Retinas* have both exhibited an overexpression of PDGF-B, which was predominantly localized within the cell bodies of the retinal neurons; and it was mostly localized to the Müller cell end-feet at the ILM with diffuse/multifocal overexpression at the NFL, GCL, and INL. Our data corroborated previous reports [47], which indicated that PDGF-B immunoreactivity was observed in Müller cell end-feet of the neural retina. The source of this PDGF-B was next investigated in a series of *in vitro* experiments in which glial cells were subjected to hypoxic conditions for 72 hours. Such treatment caused a profound increase in PDGF-B at the message and the protein levels. Taken together, these findings suggest the contribution of Müller cells to retinal PDGF-B and implicate an autocrine mechanism of PDGF-B on Müller cells. It is noteworthy that our results are in concordance with previous studies [8], which demonstrated that glial cells may utilize the elevated levels of PDGF-B to proliferate, and consequently causing RG. In this manuscript, we demonstrate that hypoxia has triggered RG within 72 hours of exposure *in vitro* [rMC-1 and R28 cells], whereas the ischemic retina has fully developed RG at P17 *in vivo* [OIR mouse model]. These findings are in concordance with previous studies [20].

Hypoxia inducible factor-1 [HIF-1] is a master regulator that controls the transcriptional activation of VEGF signaling and other hypoxia-inducible genes [53]. Like VEGF; PDGF-B is a hypoxia-regulated gene [54]. Our previous studies have revealed that YC-1 inhibits HIF-1 and other proangiogenic factors in the ischemic retinas of the OIR mouse model [38], [39], [40]. It is therefore possible that YC-1's effect on RG may be mediated through the inhibition of HIF-1-signaling, since PDGF-B protein molecule is downstream of HIF-1. Throughout our current and previous investigations, we have demonstrated that targeting hypoxia and HIF-1 signaling maybe considered as a therapeutic modality to target several downstream angiogenic molecules, such as PDGF-B, which play crucial roles in ischemic retinopathies. Moreover, sprouting angiogenesis involves collective migration processes [55]. Tip cells are distinguished by their strong expression of PDGF-B mRNA and VEGFR2 mRNA and protein, implying that tip cells may have a distinct gene expression profile [56] and regulate the coordinated processes of neovascular sprouting. These findings would be consistent with our current data, which revealed that the decrease in the length and number of neovascular sprouts in YC-1-treated retinas, were both highly associated with the downregulatory effects of YC-1 on PDGF-B expression. Taken together, this study has demonstrated that YC-1 could be exploited as valuable therapeutic modality in the treatment of RG in the ischemic retina. Antagonists of PDGFs may help to reduce scarring, but may also synergize with VEGF antagonists to reduce NV possibly through pericytes, which provide survival signals for ECs of new vessels [57]. Kinase inhibitors that block both VEGF and PDGF receptors are some of the most efficacious drugs for the treatment of ocular NV in animal models [58], [59]. Our current study has revealed that YC-1 inhibited GFAP and PDGF-B, while our previous studies have indicated that YC-1 inhibited VEGF [38], [39], [40]; such data corroborate other studies, which demonstrated that combining antagonism of PDGFs with blockade of VEGFs may be a useful strategy for treatment of ocular NV [59]. Successful inhibition of GFAP using antisense oligonucleotides has also been reported by other investigators [28], [30].

Our previous investigations have demonstrated the presence of spatial overexpression of VEGF, ET-1, iNOS, and MMP-9 in the neovascular retina of the OIR mouse model [39]. Whereas in our current study, we demonstrate a concomitant expression of GFAP and PDGF-B, which occur during ischemic retinal NV. It was reported that neoangiogenesis was associated with reactive astrogliosis and was correlated to increased reactive astrocytosis and associated VEGF expression [60]. In addition, multiple lines of evidence have demonstrated a pivotal role of the endothelin system in stimulating RG. The production of ET-1 is stimulated at injured brain sites [61], and cerebral ischemia specifically triggers astrocytes to release it [62]. Additionally, ET-1 is highly expressed in reactive astrocytes from patients who have suffered from various neurological disorders, including cerebral infarcts, and Alzheimer's disease [63]. Moreover, it was suggested that ET-R-associated pathways might represent important targets to control RG [64]. In injured nerve tissues, astrocytes become the reactive phenotype, which causes the overexpression of MMP-9 [65]. In addition, the same study has suggested that ETs are one of factors, which stimulate astrocytic MMP-9 productions. Moreover, previous studies have suggested that iNOS expression may serve as an index of RG [66], [3]. Taken together, our findings and those of others suggest a crosstalk between RG and NV. Our study demonstrates that the neuroprotective mode of YC-1's action, which blunts the ischemic insult to the retina may have similar role in protecting ischemia-induced neural damage.
